This article has been retracted.

# Anesthesia Effect of Remifentanil Combined with Propofol in Laparoscopic Cholecystectomy and Its Impact on Postoperative Cognitive Recovery

**DOI:** 10.1155/2022/9147416

**Published:** 2022-07-15

**Authors:** Wei Jiang, Jun Wang, Xin-xin Ni, Zu-chao Huang

**Affiliations:** ^1^Department of Anesthesiology, Huishan District People's Hospital, Wuxi, Jiangsu, China; ^2^Department of Anesthesiology, The Affiliated Wuxi People's Hospital of Nanjing Medical University, Wuxi, Jiangsu, China

## Abstract

**Objective:**

To investigate the anesthesia effect of remifentanil combined with propofol for laparoscopic cholecystectomy and its impact on postoperative cognitive recovery.

**Methods:**

A total of 120 patients who underwent laparoscopic cholecystectomy in our hospital from February 2019 to June 2021 were recruited and assigned into either control group or experimental group at a ratio of 1 : 1 via the random number table method. The patients in the control group were anesthetized with fentanyl combined with propofol, and the patients in the experimental group were anesthetized with remifentanil combined with propofol. The clinical basic indicators (extubation time, recovery time, breathing recovery time, and orientation recovery time), and observer's assessment of awareness/sedation (OAA/S) scores and complications were compared between the two groups.

**Results:**

There was no significant difference in extubation time between the two groups (*P* > 0.05). The postoperative wake-up time, respiratory recovery time, and orientation recovery time of the experimental group were significantly better than those of the control group (*P*  < 0.05). The OAA/S scores of the patients in the experimental group were significantly higher than those in the control group immediately after surgery, 1 h after surgery, and 3 h after surgery (*P*  < 0.05). There was no significant difference in the OAA/S scores between the two groups on the 1st day after operation (*P* > 0.05). The incidence of complications in the experimental group was significantly lower than that in the control group (*P*  < 0.05).

**Conclusion:**

Remifentanil + propofol for laparoscopic cholecystectomy patients has a significant anesthesia effect. This strategy effectively shortens the extubation, awakening, respiratory recovery, orientation recovery time of patients, and OAA/S score, suggest a minor impact on the postoperative cognitive function and state of consciousness. It has a high safety profile and thus is worthy of clinical application.

## 1. Introduction

Laparoscopic cholecystectomy is currently the mainstay for the treatment of patients with gallbladder disease. As the most effective type of minimally invasive surgery for the treatment of gallbladder disease, it excels owing to its small incision, less bleeding, fast recovery time, and high clinical efficacy [1]. Clinical studies have pointed out that in the treatment of laparoscopic cholecystectomy, treatment effects using different anesthesia methods are varying [2, 3]. Previously, clinical anesthesia for patients undergoing laparoscopic cholecystectomy majorly used fentanyl plus propofol, but the anesthesia effect yet remains unsatisfactory [4]. The disadvantages of slow metabolism and the long half-life of fentanyl are likely to prolong the recovery time of patients after surgery and the recovery time of spontaneous breathing, thereby raising the risk of a series of complications [5]. Bakan et al. [6] pointed out that the anesthesia effect of remifentanil combined with propofol in patients undergoing laparoscopic cholecystectomy produces a desirable result. Postoperative cognitive dysfunction falls into the category of neuropsychiatric complications of patients after surgery and has captured extensive attention in the academic community [6]. Evidence suggests that different anesthesia methods have an inconsistent impact on the occurrence of postoperative cognitive dysfunction. In support of the above finding, Li et al. revealed an association between anesthesia factors and the occurrence of postoperative cognitive dysfunction [7]. The principal objective of this study was to investigate the impact of remifentanil plus propofol in laparoscopic cholecystectomy on anesthesia and postoperative cognitive recovery.

## 2. Materials and Methods

### 2.1. Participants

A total of 120 patients who underwent laparoscopic cholecystectomy in our hospital from February 2019 to June 2021 were recruited and assigned to either the control group or experimental group at a ratio of 1 : 1 via the random number table method. The control group included 37 males and 23 females; aged 60–81 years, mean age (69.28 ± 5.32) years; course of disease 1–3 years, mean course of disease (2.31 ± 0.46) years; ASA classification: 41 cases of grade I, 19 cases of grade II. In the experimental group, there were 39 males and 21 females; aged 60–80 years, with an average age of (69.17 ± 5.30) years; the course of the disease was 1–4 years, with an average course of (2.39 ± 0.52) years; ASA classification: 40 cases were grade I and 20 were grade II. This study has been approved by the Clinical Trial Ethics Committee of our hospital prior to the enrollment, and all patients and their families voluntarily participated in this study.

### 2.2. Inclusion and Exclusion Criteria

Inclusion criteria: (1) the patients had good compliance; (2) the patients have not received other surgery or anesthesia in recent years. Exclusion criteria: (1) patients with other organ diseases; (2) patients who are allergic to the study drug; (3) patients with communication disorders.

### 2.3. Methods of Anesthesia

Twenty minutes before surgery, 0.1 g of phenobarbital + 0.5 mg of atropine were intramuscularly injected into the two groups. After the patient entered the operating room, their vital signs were closely monitored, they were given mask oxygen, and intravenous access was established. The patients in the control group were anesthetized with fentanyl combined with propofol. The essence is intravenous injection of propofol 1.3 mg/kg + fentanyl 3.5 *μ*g/kg + atracurium cissulfonate 0.5 mg/kg. They were then intubated and mechanically ventilated. Fentanyl 2.5 *μ*g/kg was administered intravenously to the patient 2 min before the surgical procedure. During the operation, anesthesia was maintained with 40 *μ*g/kg/min of propofol, and the propofol was stopped after the surgical treatment [8]. The patients in the experimental group were anesthetized with remifentanil combined with propofol. The essence is intravenous injection of propofol 1.3 mg/kg + remifentanil 2 *μ*g/kg + atracurium cissulfonate 0.5 mg/kg. They were then intubated and mechanically ventilated. During the operation, 40 *μ*g/kg/min of propofol and 0.4 *μ*g/kg/min of remifentanil were used to maintain anesthesia, and the remifentanil and propofol were stopped after the surgical treatment [9].

### 2.4. Outcomes

1. Basic clinical indicators were recorded by medical staff in our hospital including extubation time, recovery time, breathing recovery time, and orientation recovery time.
2. The observer's assessment of awareness/sedation (OAA/S) score [10] was used to evaluate the state of consciousness of patients immediately after operation, 1 h after operation, 3 h after operation, and 1 d after operation. The higher the OAA/S score, the better the patient's state of consciousness. 5 points indicate rapid response to normal shouting; 4 points indicate indifferent response to normal shouting; 3 points indicate responding only to loud shouts; 2 points indicate responding only to gentle shaking; 1 point indicates no response to mild shaking; 0 point indicates no response to squeezing the trapezius.
3. Complications include nausea and vomiting, respiratory depression, restlessness, and urinary retention.

### 2.5. Statistical Analysis

Measurement data were expressed as the mean ± standard deviation, and count data were expressed as case or rate. Statistical analysis was performed using SPSS 22.0 (IBM, Armonk, NY, USA). Differences between measurement data and count data were compared using Student's *t*-test and chi-square test, respectively. A *P* value <0.05 was considered statistically significant.

## 3. Results

### 3.1. Baseline Data

There was no significant difference in baseline data between the two groups of patients (*P*  > 0.05), as shown in Table 1.

### 3.2. Basic Clinical Indicators

There was no significant difference in extubation time between the two groups (*P*  > 0.05). The postoperative wake-up time, respiratory recovery time, and orientation recovery time of the experimental group were significantly better than those of the control group (*P* < 0.05) (see Table 2).

### 3.3. OAA/S Score

The OAA/S scores of the patients in the experimental group were significantly higher than those in the control group immediately after surgery, 1 h after surgery, and 3 h after surgery (*P* < 0.05). There was no significant difference in the OAA/S scores between the two groups on the 1st day after operation (*P*  > 0.05) (see Table 3).

### 3.4. Complications

The incidence of complications in the experimental group was significantly lower than that in the control group (*P* < 0.05, Table 4).

## 4. Discussion

Despite the widespread availability of laparoscopic cholecystectomy, it is associated with cognitive dysfunction in elderly patients [11]. The major contributor is the declined functions of the body in elderly patients, leading to a decreased ability in metabolizing anesthetic drugs and increasing the risk of postoperative cognitive dysfunction [12]. Patients with postoperative cognitive dysfunction show manifestations of disorders concerning orientation, memory, and abstract thinking, as well as social activity. In addition to hindering postoperative recovery and prolonging the hospitalization stay, it imposes a substantial medical cost burden on patients [13]. This suggests the potential value of providing options to treat postoperative cognitive dysfunction. There remains an urgent need to explore an anesthesia strategy that has a mild impact on postoperative cognitive function [14]. Propofol is an ultra-short-acting intravenous anesthetic with high lipid solubility and almost insoluble in water. Due to its rapid onset of action, rapid and stable recovery of patients, with slight discomfort after recovery, it has been well-recognized in clinical practice [15]. The molecule of the new ultra-short-acting opioid, remifentanil, contains an ester bond, and its drug is mainly hydrolyzed by nonspecific esterases, resulting in the drug metabolism insusceptible to liver and kidney functions [16]. Additionally, it has the advantages of a small volume of distribution, rapid onset of action, fast elimination, and no accumulation in the patient's body [17], which makes the drug suitable for continuous infusion administration. Even if it is used in large quantities for a long time, it will not lead to the residual effect of the drug after stopping the drug, with no impact on the recovery of patients after surgery [18].

In this study, we found that the postoperative wake-up time, respiratory recovery time and orientation recovery time of the experimental group were significantly better than those of the control group. In addition, the OAA/S scores of the patients in the experimental group were significantly higher than those in the control group immediately after surgery, 1 h after surgery, and 3 h after surgery; there was no significant difference in the OAA/S scores between the two groups on the 1st day after operation. Encouragingly, the incidence of complications in the experimental group was significantly lower than that in the control group. The possible reasons may be that compared with other opioids, remifentanil is more effective with the advantages of fast onset and long anesthesia time, and the characteristics of fast elimination and no accumulation in the patient's body, which makes the drug practical in large quantities for a long time. And the combined use of remifentanil and propofol can exert a good synergistic effect, and this can further improve the anesthesia effect of patients [19, 20]. The underlying mechanism is that the use of propofol combined with lipopolysaccharide has an effect on A549 cells, and propofol can block LPS-induced related autophagy proteins. Opioid receptors are a family of *G* protein-coupled receptors with several hundred genes in the human genome. Its opioid receptor protein has a variety of active structures. Many regulatory proteins also affect opioids, which in turn modulate receptor activity and structure. Calmodulin, Go/Giot proteins, kinases and other types of regulatory proteins, and multidomain proteins or chaperones can also affect the pharmacological properties of opioid receptors. Remifentanil belongs to the current new type of opioid receptor agonist, with short action time, rapid onset of action, rapid recovery, and strong controllability. Also, the anesthesia drugs are eliminated faster in patients using remifentanil combined with propofol, which minimizes the impact of anesthetic drugs on the cognitive function and state of consciousness [21].

In addition, the traditional Chinese medicine acupuncture treatment of diseases began with the legend of “Fuxi made nine needles,” and the classical medical books “Huangdi Neijing” and “Acupuncture and Moxibustion A and B Classic.” Acupuncture can treat a variety of diseases, but there is no clear record that anesthesia can be performed. According to the fact that acupuncture can relieve pain, people boldly proposed the idea of using acupuncture for “anesthesia” in conjunction with surgery. The selection of acupuncture points according to the surgical site and the principle of meridians is the main method that must be followed [22]. For example, thyroid surgery and tonsil surgery generally select two acupoints of Hegu and Neiguan on both sides, while thoracotomy lobectomy initially selects more than 20 acupoint pairs based on the principle of meridians. Subsequently, the number of acupuncture points was reduced to about 5 pairs. The practice has also found that the selection of acupuncture points is not completely consistent with the correlation between meridians and collaterals, and practical experience should be the mainstay.

However, there are a few limitations to consider. Our study was conducted on a relatively homogenous population; the sample size analyzed is relatively small, which reduces the reliability of the study. To overcome these limitations, future research will still need to potentially include a larger sample size with heterogenous backgrounds and environments.

To sum up, remifentanil + propofol for laparoscopic cholecystectomy in patients has a significant anesthesia effect. This strategy effectively shortens the extubation, awakening, respiratory recovery, and orientation recovery time of patients, and OAA/S score, suggesting a minor impact on the postoperative cognitive function and state of consciousness. It has a high safety profile and thus is worthy of clinical application.

## Figures and Tables

**Table 1:** Baseline data.

	Control group (*n* = 60)	Experimental group (*n* = 60)	*t* or *x*^2^	*P* value
Gender				
Male	37	39	0.144	0.705
Female	23	21		
Age (year)	$\bar{X}\pm s$	$\bar{X}\pm s$		
Mean age (year)	69.28 ± 5.32	69.17 ± 5.30	0.113	0.91
Course of disease (year)	$\bar{X}\pm s$	$\bar{X}\pm s$		
Mean course (year)	2.31 ± 0.46	2.39 ± 0.52	−0.893	0.374
ASA				
Grade I	41	40	0.038	0.845
Grade II	19	20		

**Table 2:** Comparison of basic clinical indicators ($\bar{X}\pm s$).

Groups	Extubation time (min)	Wake-up time (min)	Breathing recovery time (min)	Orientation recovery time (min)
Control group (*n* = 60)	8.34 ± 1.27	8.57 ± 0.76	6.24 ± 0.46	12.21 ± 1.44
Experimental group (*n* = 60)	8.24 ± 1.25	6.40 ± 0.43	2.11 ± 0.20	8.09 ± 1.03
*t*	0.435	19.249	63.778	18.026
*P* value	0.664	<0.001	<0.001	<0.001

**Table 3:** OAA/S score comparison ($\bar{X}\pm s$).

Groups	Immediately after operation	1 h after operation	3 h after operation	1 d after operation
Control group (*n* = 60)	3.30 ± 0.25	3.94 ± 0.38	4.24 ± 0.50	4.66 ± 0.61
Experimental group (*n* = 60)	3.55 ± 0.27	4.33 ± 0.36	4.59 ± 0.58	4.75 ± 0.64
*t*	−5.263	−5.771	−3.54	−0.788
*P* value	<0.001	<0.001	0.001	0.432

**Table 4:** Comparison of complications.

Groups	Nausea and vomiting	Respiratory depression	Restless	Urinary retention	Incidence (%)
Control group (*n* = 60)	2	2	3	1	8 (13%)
Experimental group (*n* = 60)	1	0	1	0	2 (3%)
*X* ^2^	—	—	—	—	3.927
*P* value	—	—	—	—	0.048

## Data Availability

No data were used to support this study.
